# Foliar application of potassium and moringa leaf extract improves growth, physiology and productivity of kabuli chickpea grown under varying sowing regimes

**DOI:** 10.1371/journal.pone.0263323

**Published:** 2022-02-10

**Authors:** Sohail Irshad, Amar Matloob, Shahid Iqbal, Danish Ibrar, Zuhair Hasnain, Shahbaz Khan, Nabila Rashid, Muhammad Nawaz, Rao Muhammad Ikram, Muhammad Ashfaq Wahid, Abdulrahman Al-Hashimi, Mohamed S. Elshikh, Zeng-Hui Diao

**Affiliations:** 1 Department of Agronomy, MNS-University of Agriculture, Multan, Pakistan; 2 Department of Plant and Environmental Sciences, University of Copenhagen, Copenhagen, Denmark; 3 National Agricultural Research Center, Islamabad, Pakistan; 4 Department of Agronomy, PMAS- Arid Agriculture University, Rawalpindi, Pakistan; 5 Department of Botany, University of Agriculture, Faisalabad, Pakistan; 6 Department of Agricultural Engineering, KFUEIT, Rahim Yar Khan, Pakistan; 7 Department of Agronomy, University of Agriculture, Faisalabad, Pakistan; 8 Department of Botany and Microbiology, College of Science, King Saud University, Riyadh, Saudi Arabia; 9 Guangdong Provincial Engineering and Technology Research Center for Agricultural Land Pollution Prevention and Control, Zhongkai University of Agriculture and Engineering, Guangzhou, China; Anhui Agricultural University, CHINA

## Abstract

Chickpea (*Cicer arietinum* L.) is of prime importance because of vital source of protein as major food legume. Globally, it is cultivated on large area to meet dietary requirements of humans. Climatic extremes (erratic rainfall, extreme high and low temperature) are key restrains for its production. Optimum sowing time is considered as an important factor to address climatic variations and to attain maximum yield. Foliar application of potassium (K) has also been reported to increase resistance against abiotic stresses. Similarly, exogenous application of plant based growth substances (bio-stimulants) like moringa leaf extract (MLE) are extensively used to enhance productivity of field crops. Therefore, current study was planned to evaluate the impact of foliar applied K and MLE on growth, physiology and productivity of kabuli chickpea grown under varying sowing dates. There were two sowing dates (normal sown; November 15 and late sown; December 15, 2020). Experiment was comprised of treatments i.e. control, water spray, foliar application of K at 1%, foliar application of MLE at 3% and combined application of K and MLE. Foliar applied K and MLE significantly improved physiological, biochemical and yield attributes of kabuli chickpea cultivated under normal and late sown conditions. Increase in growth and yield attributes like plant height, number of nodules per plant, nodules dry weight, branches and pods per plant, 100- grain weight, biological and grain yield were recorded in case of combined foliar application of K and MLE in normal and late sown chickpea. Maximum improvement in gas exchange attributes (stomatal conductance and transpiration rate), chlorophyll contents, antioxidants (catalase, superoxide dismutase and ascorbate peroxidase) and osmolytes (proline) were recorded with combined application of K and MLE in both sowing dates. Thus, combined applied K and MLE can be used to enhance productivity of kabuli chickpea.

## Introduction

Pulses have emerged as the most important crops which have been grown by human beings since time immortal. They are also known as leguminous food crops throughout the globe. Cultivation of pulses play very crucial role in the economy of the country. Chickpea (*Cicer arietinum*) in one of the most economical important food legumes cultivated round the world [1] as it plays vital role in human nutrition [2]. It is rich source of protein (21%), carbohydrates (61%) and oil (2.2%) [3] and classified as highly nutritious and healthy food [4]. It helps in improving and sustaining soil fertility by nitrogen (N) fixation [5]. However, the productivity of chickpea is not sufficient to fulfill the protein requirement for ever increasing masses [6,7]. Its production is limited by a number of abiotic (frost damage, drought, terminal heat etc.) and biotic (diseases and weeds) stresses [8]. Most importantly, unpredictable climate change is the major constraint for chickpea production as it increases the frequency of drought and temperature extremes i.e. high (> 30°C) and low (< 15°C) temperatures which reduces grain yields considerably [9,10].

Sowing time and techniques of any crop are mainly responsible for maximum growth and yield because it is an interaction of variety with its environment [11,12]. Flowering is an important phenomenon which has crucial role in final yield of crop and its development is more prone to environmental variations. Increase in temperature at flowering stage of chickpea is main cause of flower abortion [13]. Temperature is one of the critical factor causes flower abortion of chickpea when it exceeds more than 35ºC [14]. Sowing of chickpea at optimum time outcomes timely initiation of flowering that minimize the impact of terminal heat and early cold stress resultantly better growth and development of chickpea plants [8]. Early sown chickpea results in lodging of crop, more disease incidence and drought stress at grain filling stage while late sown chickpea is more prone to insect attack, less vegetative cover and reduced water use efficiency [15]. Farmers have wrong perception that being legume crop, there is no nutritional requirements of chickpea and it is grown on marginal lands without any proper nutrition. Proper nutrition has significant role in improving growth and yield of pulses [16].

A set of physio-chemical, biological and integrated approaches is available for reducing yield losses [17–19]. Among them, the use of organic (biostimulants) and inorganic (nutrient and chemical agents) growth stimulators are considered viable approaches to compensate yield losses [19,20]. Biostimulants are natural growth enhancers that stimulate crop yield via enhanced nutrient uptake and efficiency, improved tolerance to biotic and abiotic stresses and enhancement of the rhizospheric activities [21]. Natural sources like seaweed extracts, protein hydrolysates and amino acids, humic acid, fulvic acid, complex organic materials, chitin and chitosan derivatives, microbial inoculants, biochar and plant extracts are the most commonly used biostimulants in agriculture [21–23]. *Moringa oleifera* leaf extract, sorghum water extract and mulberry water extracts are commonly used growth enhancers when applied as a seed priming agent and/or foliar spray [24,25]. It has been scientifically proven that they positively modify plant growth and production with alterations in metabolic processes under different cultivation practices [25–28]. Rehman *et al*. [29] also reported that application of plant growth promoters in combination with mineral elements improved the early growth, better establishment of seedlings and other yield contributing factors.

Moringa, among all the naturally occurring plant growth stimulants, has received enormous attention from the scientific community because of its rich source of growth hormones (zeatin), antioxidants, vitamins and mineral nutrients in its leaves [30]. Rashid *et al*. [31] and Makawita *et al* [32] stated that foliage application of biostimulants i.e. sea weed extract, is good source of nutrient to uplift the crop productivity. Potassium (K) is major element which has important role in many plant processes [33] and its application is usually abandoned causing nutrient imbalances that reduce crop yields [34]. Foliar feeding of K improves enzymatic systems, water use efficiency, protein formation, nitrogen assimilation and photosynthesis [35]. Kumar and Rao [36] reported that an increase in the production of pulses was observed when K was applied at 20–40 kg K ha^-1^. Younas *et al*. [37] also reported that external application of chemicals induces resistant against the diseases in field crops. Currently, farmers are conscious about inorganic fertilization to increase crop production and maintaining soil fertility but there is need to promote the use of organic fertilizers and explore safe, alternative and natural plant based nutrients [38–40]. Tabaxi *et al*. [41] also concluded that organic fertilization is also responsible for quantity as well as quality of produce cultivated under field conditions. Zahid *et al*. [42] confirmed that combined application of inorganic fertilizer like urea and poultry had prominent impact on plant height, leaf area, number of leaves per plant, fruit weight and postharvest quality of cucumber. Application of mineral elements in combination with organic compounds is a good agronomic practice to increase quality of field crops [43,44].

Foliar feeding or exogenous application of nutrients and organic compounds is very effective method to meet nutritional deficiencies, transmission of nutrients, quick and effectual use of nutrients and reduced leaching & fixation losses of nutrients [25,45]. Under water deficit conditions, foliar feeding of nutrients results in higher uptake of nutrients than soil application [46]. Number of studies has shown that foliar application can boost yield up to 12–25% and 90% of the nutrient applied is consumed by the plant [47]. Foliar feeding of nutrients at flowering and seed development is gaining extensive attention to increase seed yield in pulses. Hakoomat *et al*. [48] reported among various factors, weed management, latest production technology, high yielding varieties and balanced nutrition are of prime importance. Khan *et al*. [28] that application of MLE either alone or/and in combination with inorganic growth enhancer is responsible for improved growth and productivity of cereal crops particularly wheat as MLE application plays its role in crops to maintain water balance, membrane stability, boosts antioxidant activity, increase production of secondary metabolites and enhance crop performance [25,27,40]. Less information is available on foliar application of MLE in combination with potassium on growth and productivity of chickpea. Keeping in view the above rational, current study was planned to evaluate the impact of foliar application of K and MLE either sole or/and in combination on growth and productivity of chickpea cultivated under varying sowing regimes (normal sown and late sown chickpea).

## Materials and methods

### Experimental particulars

The planned study was conducted at the Research Area, MNS-University of Agriculture, Multan, during rabi season of 2020–21. The experiment was laid out in randomized complete block design (RCBD) with split plot arrangement having three replications with a net plot size of 20 m^2^ (5m × 4 m). Experimental soil was loam in texture and other details of physic-chemical attributes are presented in Table 1. Seedbed was thoroughly prepared by ploughing followed by planking after soaking irrigation. Seed of kabuli gram, cv. Noor 2013, was obtained from Ayub Agricultural Research Institute, Faisalabad-Pakistan. Crop was sown with the help of hand drill in 45 cm spaced rows and plant spacing of 15 cm using seed rate of 60 kg ha^-1^. Crop was sown on November 15, 2020 was considered as normal sowing while sown on December 15, 2020 was considered as late sowing.

**Table 1:** Physical and chemical properties of experimental soil.

Soil Analysis	Unit	Value
**Physical Characteristics**		
Sand	%	39
Silt	%	42
Clay	%	19
Texture Class		Loam
**Chemical Characteristics**		
pH		7.9
EC	dS m^-1^	5.21
Nitrogen	me/l	0.0622
Available phosphorus	ppm	7.9
Potassium	me/l	76
Organic matter	%	1.01

The weather data, including maximum temperature, minimum temperature, mean temperature, relative humidity and rainfall, are presented in Fig 1. Fertilizers were applied at 32 and 85 kg ha^-1^ of phosphorus and nitrogen, respectively. All phosphorus was applied at the time of planting while nitrogen was applied in two splits, half the dose was applied at sowing time while the remaining was applied at 1^st^ irrigation after sowing of 45 days. Total three irrigations, at suitable intervals, were given till maturity. Other agronomic practices were kept normal and uniform. Necessary plant protection measures were adopted to keep crop free of weeds, insects and diseases.

**Fig 1:** Weather data of the experimental station during 2020–2021 growing season of crop.

### Treatments plan and extract preparation

Study was planned with two sowing dates (normal and late) and comprised of following treatments i.e. control, water spray, foliar application of K at 1%, foliar application of MLE at 3% and combined foliar application of K and MLE. All the treatments were foliar applied at flowering stage. Source of K was KCl and for 3% MLE preparation protocol was adopted as prescribed by Khan *et al*. [28]. For MLE extraction, healthy, fresh and mature leaves from moringa tree were collected. Leaves were thoroughly rinsed with tap water and were placed in refrigerator for a night. Extract was prepared using locally assembled machine and dilution of extract was made consuming distilled water to prepare 3% solution.

### Chlorophyll pigment and gas exchange attributes determination

Data regarding chlorophyll pigment and gaseous exchange attributes were recorded after one week of treatment’s application. Chlorophyll contents of leaves were measured using SPAD (502 plus) and data were recorded from three tagged plants in each treatment plot and mean value was calculated. For data collection, flag leaf was used for estimation stomatal conductance (*gs*) (mmol m^-2^s^-1^) and transpiration rate (*E*) (mmol H_2_O m^-2^s^-1^) were assessed by following the standard protocols prescribed by Long *et al*. [49] using an infrared gas analyzer (IRGA) *ADC Bio-Scientific Ltd*. *LI-6400* portable device.

### Enzymatic and quality attributes

Data regarding antioxidant enzymatic activity and osmolytes were also determined after one week of treatment’s application. The SOD activity was measured according to Giannopolotis and Ries [50]. The activity of CAT was recorded by using spectrophotometer with the performance set according to Chance and Maehly [51]. Ascorbate peroxidase (APX) activity was estimated according to Nakano and Asada [52] with slight modification. Free proline in leaf tissues was appraised by following the protocol of Bates *et al*. [53]. The K^+^ concentration in grain was measured by using flame photometer (Sherwood, UK, Model 360) according to the standard procedure of USDA, Laboratory Staff [54]. For protein determination, seed nitrogen was analyzed using Kjeldahl method [55]. Percent crude protein was calculated using acid based titration and volume of acid used was multiplied by 6.25.

### Agronomic and yield attributes

Plant height and number of branches per plant were recorded at maturity. Plant height was measured from three randomly selected plants with the help of meter rod and their branches were counted manually. Data regarding number of nodules were recorded at 60 days after sowing, for this purpose three randomly plants were uprooted carefully, washed and their nodules were separated from roots and counted. These nodules then oven dried till constant weight to get the data of nodules dry weight by using electronic weighing balance. For the estimation of number of pods per plant, five plants were randomly selected from each experimental unit after harvesting and their pods were counted. At maturity, whole plants with grains were harvested from 1 m^2^ area, sun dried and weighed to get biological yield in kg and later converted to kg ha^-1^. 100-grain weight was recorded by weighing 100 grains from each experimental unit by using electronic weighing balance. Grain yield was determined by harvesting area of 1 m^2^ from each plot, weighed and then converted in kg ha^-1^. Harvest index was calculated as it is the ratio of grain yield to total (above ground) biological yield expressed in percentage.

Harvestindex=Grainyield/Biologicalyield×100

### Statistical analysis

Compiled data related to growth, physiology and productivity were examined statistically using statistical package “Statistic 8.1”. Fisher’s analysis of variance technique (ANOVA) was used for testing significance of collected data. For graphical presentation and estimation of standard errors Microsoft excel was used. Difference among treatment means was equated by employing HSD, Tukey’s test at the level of 5% probability [56].

## Results

Significant levels of growth, gas exchange, osmolytes, enzymatic antioxidants activity, yield and quality parameters in response to foliar applied K and MLE in normal and late sown kabuli chickpea is presented in Table 2. Data regarding number of nodules, nodules dry weight and plant height are presented in Table 3. Highest value of nodules per plant were observed in normal sowing followed by late sowing. Maximum nodules per plant were observed in combined application of K and MLE followed by MLE, K, water spray and control while interaction of foliar treatments and sowing dates was non-significant. In case of nodules dry weight per plant, similar trend regarding sowing dates was observed while maximum value of nodules dry weight was observed in combined application of K and MLE which was statistically similar to sole application of MLE and minimum value was observed in control and interaction was non-significant. Regarding sowing dates, highest value of plant height was observed in case of normal sowing followed by late sowing. Regarding treatments, maximum value of plant height was observed in case of combined foliar application of MLE and K which is statistically similar to sole application of MLE and minimum value was observed in control (Table 3). Interaction of sowing dates and foliar treatments for plant height was statistically non-significant (Table 2).

**Table 2:** Mean sum of squares of growth, physiological and yield parameters in response to foliar applied K and MLE in normal and late sown kabuli chickpea.

SOV	Chl.	*E*	*Gs*	NdPP	NdDW	PH
Treatments (T)	599.7**	1.102**	367.4**	3.883^NS^	9.653*	113.2**
Sowing dates (S)	34.11*	5.241*	2231**	8.533*	297.1**	785.4**
T × S	2.53^NS^	0.073^NS^	46.14**	0.616^NS^	0.470^NS^	2.825^NS^
	BPP	PP	HGW	BY	GY	HI
Treatments (T)	31.88**	198.1**	8.878**	263987 **	32982**	19.49 **
Sowing dates (S)	229.6**	554.7**	2.465**	2538103**	1637069**	167.2**
T × S	3.217^NS^	1.783^NS^	0.201**	80988**	47326**	3.743**
	CAT	SOD	APX	Proline	GPC	GKC
Treatments (T)	43.84**	63.82**	14.89**	5.33**	4.652**	7.518**
Sowing dates (S)	34.35*	63.95*	34.77*	14.26**	1.875*	1.008^NS^
T × S	21.56**	40.38**	9.05**	0.017^NS^	0.062^NS^	0.044^NS^

SOV = Source of variance, Chl = Chlorophyll, *E* = Transpiration rate, *gs* = stomatal conductance, NdPP = Nodules per plant, NdDW = Nodules dry weight, PH = Plant height, BPP = Branches per plant, PP = Pods per plant, HGW = 100-grain weight, BY = Biological yield, GY = Grain yield, HI = Harvest index, CAT = Catalase, SOD = Superoxide dismutase, APX = Ascorbate peroxidase, GPC = Grain protein contents, GKC = Grain potassium contents NS = Non-significant,

* = Significant at P ≤ 0.05,

** = Significant at P ≤ 0.01.

**Table 3:** Impact of foliar applied potassium and moringa leaf extract on number of nodules per plant, nodules dry weight (mg) and growth and plant height (cm) of normal and late sown kabuli chickpea.

Treatments	Nodules per plant			Nodules dry weight (mg)			Plant height (cm)		
	NS	LS	Mean (T)	NS	LS	Mean (T)	NS	LS	Mean (T)
Control	11.33	10.66	11.00A	38.66	32.43	36.55B	48.80	39.53	44.16C
Water spray	11.66	10.66	11.16A	39.00	33.50	36.25AB	50.46	42.13	46.30C
K 1%	13.33	11.33	12.33A	40.66	34.53	37.60AB	56.63	45.50	51.06B
MLE 3%	13.00	11.66	12.33A	41.33	34.33	37.83AB	58.53	46.96	52.75AB
K + MLE	13.00	12.66	12.83A	42.00	35.40	38.70A	59.33	48.96	54.40A
Mean (S)	12.46A	11.40B		40.33A	34.04B		54.85A	44.62B	
**HSD**	S = 0.574, T = NS, S×T = NS			S = 3.012, T = 2.987, S×T = NS			S = 2.29, T = 2.389, S×T = NS		

Means sharing the same letter did not differ significantly at P = 0.05, MLE = Moringa leaf extract, K = Potassium, S = Sowing date, T = Foliar treatments

Late sowing of chickpea significantly reduced the number of branches per plant as maximum branches were observed in normal sown crop (Table 4). Regarding foliar treatment, highest number of branches per plant were attained by combined application of K and MLE which was statistically similar to sole application of MLE followed by K. Minimum value was observed in case of control and interaction was non-significant. In case of number of pods per plant, similar trend was observed regarding sowing regimes. In case of foliar treatments, application of K+MLE produced maximum pods per plant followed by sole application of MLE and K. Highest value of 100-grain weight was attained in normal sowing of chickpea followed by late sowing. In case of foliar treatments, highest 100-grain weight was observed in combined application of K and MLE which was statistically similar to MLE followed by K. Interaction between sowing dates and foliar treatments was also found statistically significant. Combined application of K and MLE was responsible for maximum 100-grain weight of chickpea under normal sowing conditions.

**Table 4:** Impact of foliar applied potassium and moringa leaf extract on number of branches per plant, number of pods per plant, and 100-grain weight of normal and late sown kabuli chickpea.

Treatments	Branches per plant			Pods per plant			100-grain weight (g)		
	NS	LS	Mean (T)	NS	LS	Mean (T)	NS	LS	Mean (T)
Control	18.33	13.33	15.83B	45.33	38.33	41.83D	25.16e	24.36f	24.76E
Water spray	18.66	14.00	16.33B	49.00	39.33	44.16D	25.50e	25.26e	25.38D
K 1%	19.33	15.33	17.33B	52.66	44.66	48.66C	26.66cd	26.55d	26.60C
MLE 3%	23.00	16.66	19.83A	56.33	47.00	51.66B	27.51b	26.66cd	27.09AB
K + MLE	25.00	17.33	21.16A	60.66	51.66	56.16A	28.15a	27.28bc	27.71A
Mean (S)	20.86A	15.33B		52.80A	44.20B		26.60A	26.02B	
**HSD**	S = 2.29, T = 2.389, S×T = NS			S = 3.107, T = 4.694, S×T = NS			S = 0.199, T = 0.375, S×T = 0.672		

Means sharing the same letter did not differ significantly at P = 0.05, MLE = Moringa leaf extract, K = Potassium, S = Sowing date, T = Foliar treatments.

Data regarding biological yield, grain yield and harvest index are presented in Table 5. In case of biological yield there was significant effect of foliar treatments and sowing dates as well as their interaction. Highest biological yield was attained in normal sowing of chickpea crop followed by late sowing. In case of foliar treatments, maximum value was in case of K+MLE which was statistically similar to MLE and minimum value was observed in case of control. Under interaction circumstances, combined application of K and MLE produced highest biological yield under normal sowing conditions. In case of grain yield, highest value was observed in case of normal sowing followed by late sowing. Regarding foliar treatments, maximum value was observed in case of K+MLE application followed by MLE and K. Interaction between sowing dates and foliar treatments was also recorded significant. Interaction of sowing dates and foliar treatments regarding harvest index (HI) was recorded statistically significant. Maximum value of HI was observed by combined application of K and MLE under late sown conditions.

**Table 5:** Impact of foliar applied potassium and moringa leaf extract on biological yield (kg/ha), grain yield (kg/ha) and harvest index of normal and late sown kabuli chickpea.

Treatments	Biological yield (kg/ha)			Grain yield (kg/ha)			Harvest index (%)		
	NS	LS	Mean (T)	NS	LS	Mean (T)	NS	LS	Mean (T)
Control	3136.0e	2803.0g	2969.5E	1800.3d	1528.7ef	1664.5D	42.59e	45.46c	44.02B
Water spray	3255.0d	2854.0dg	3054.5D	1904.3c	1549.7e	1727.0C	41.49f	45.70c	43.59C
K 1%	3502.7c	2965.7f	3234.2C	1916.3c	1509.3f	1712.8C	45.29c	49.10b	47.19A
MLE 3%	3767.3b	3007.7f	3387.5B	2107.0b	1499.7f	1803.3B	44.07d	50.14a	47.11A
K + MLE	3899.0a	3021.0f	3460.0A	2197.3a	1502.0f	1849.7A	43.64d	50.28a	46.96A
Mean (S)	3512.0A	2930.3B		1985.1A	1517.9B		43.41B	48.13A	
**HSD**	S = 37.88, T = 33.20, S×T = 55.817			S = 33.39, T = 17.85, S×T = 74.06			S = 0.537, T = 0.318, S×T = 1.1978		

Means sharing the same letter did not differ significantly at P = 0.05, MLE = Moringa leaf extract, K = Potassium, S = Sowing date, T = Foliar treatments.

Data regarding impact of foliar applied K and MLE on chlorophyll contents and transpiration rate are presented in Fig 2. Highest concentration of chlorophyll was observed in normal sowing followed by late sowing. Combined application of K and MLE produced maximum concentration of chlorophyll which was statistically similar to alone application of MLE followed by K while minimum in control treatment. Fig 2 also represents the data regarding transpiration rate which was statistically significant. Normal sowing of chickpea represented highest value of transpiration rate followed by late sowing while, in case of foliar treatment, highest value was observed in case of K+MLE which was statistically similar to MLE followed by K. Data regarding stomatal conductance (*gs*) and ascorbate peroxidase (APX) activities are given in Fig 3. Maximum *gs* was recorded under normal sown by combined application of K and MLE followed by alone MLE and K under normal sowing. While lowest *gs* was observed in control treatment under late sowing.

**Fig 2:** Impact of foliar applied K and MLE on chlorophyll contents and transpiration rate of early and late sown kabuli chickpea.

**Fig 3:** Impact of foliar applied K and MLE on stomatal conductance and ascorbate peroxidase activity of early and late sown kabuli chickpea.

Maximum activities of APX recoded under late sowing of chickpea by combined application of K and MLE followed by alone application MLE under late sowing (Fig 3). Fig 4 depicted the data regarding the activities of catalase (CAT) and superoxide dismutase (SOD) in chickpea cultivated under normal and late sown conditions in response to application of K and MLE. The interaction of foliar treatments and sowing date was observed statistically significant (Table 2). Maximum activity of CAT was analyzed by combined application of K and MLE under late sown conditions followed by alone MLE application under same sowing conditions. Minimum activity of CAT was recorded under control treatment. SOD activity was also recorded highest by combined application of K and MLE under late sown conditions.

**Fig 4:** Impact of foliar applied K and MLE on CAT and SOD activities of early and late sown kabuli chickpea.

Data regarding leaf proline, grain protein and grain potassium are expressed in Fig 5. All the foliar treatments significantly improved the proline concentration in leaf but maximum improvement was recorded by the combined application of K and MLE. In case of sowing regimes, maximum proline activity was analyzed under normal sowing of chickpea as compared to late sowing. Highest value of protein in grain was observed in case of normal sowing as compared to late sowing. Combined application of K and MLE produced maximum K concentration in chickpea grains followed by alone application of K. Minimum K concentration was found under control and water spray application. Late sowing of chickpea significantly reduced the K concentration in chickpea grains (Fig 5).

**Fig 5:** Impact of foliar applied K and MLE on leaf proline (a), grain protein (b) and grain potassium contents of early and late sown kabuli chickpea.

## Discussion

Results of current study revealed that combined application of K and MLE increased gas exchange, biochemical attributes, growth and yield of normal and late sown kabuli chickpea. Significant increase in different growth and yield attributes like plant height, nodules per plant, nodules dry weight, branches and pods per plant was found by combined application of K and MLE while in case of sowing dates normal sowing performed better than late sowing. Number of scientists put forth the impact of sowing dates on yield and yield related attributes in chickpea [57]. Timely sowing resulted in better growth and yield while late sown chickpea after 15^th^ November, ensued poor stand and short life span because of adverse climatic conditions [58]. Harvesting period and weather conditions had a significant impact on produce as well as its quality [59]. Our findings are in agreement with Kabier *et al*. [60] who reported an increase in plant height in normal sown chickpea due to increased vegetative growth because of promising weather conditions as compared to late sowing. Similar results were testified by Mansur *et al*. [61] who reported that maximum number of branches per plant in case of early sown (15 November) and lowest branches of chickpea were in late sowing (30 November) were observed. Number of pods per plant is an important yield contributing factor which was also affected by sowing dates. Highest pods were noted in early sowing as compared to late sowing. Imran *et al*. [62] reported that exogenous application of nitrogenous fertilizer increased the plant height, grains per cob and economical yield of maize hybrids. Our findings are in line with Dixit *et al*. [63] and Siddique and Sedgley [64] who reported a decrease in number of pods per plant in case of late sown chickpea. Regarding foliar applied treatments MLE alone and in combination with K significantly affected yield attributes in current study. Foliar application of MLE can improve crop performance by enhancing water status, membrane stability, enzyme system and growth of plant [65]. Foliar applied K has advantage of correcting K deficiency quickly in plant in late sowing as compared to soil application [66] as it involved in many plant physiological processes, enzyme activation, assimilation and photosynthesis and has direct impact on productivity of crop [67]. Farooq *et al*. [68] confirmed that foliar applied brassica water extract significantly improved the seedling characteristics like shoot/root biomass, shoot/root length and number of leaves in chickpea and yielded maximum. Findings of our study affirmed the reports of Asif *et al*. [69] who reported an increase in plant height, nodules per plant, number of secondary branches, pods per plant and grain yield chickpea (CM 98) by K application at varying rates. Ganga *et al*. [70] also confirmed our findings. Combined application of K and MLE improved overall growth and yield attributes which might be due to maximum availability of nutrients, growth promoting hormones that increased enzymatic activity, photosynthetic rate and various biochemical processes [71]. Our findings are in accordance with Yasmeen *et al*. [72] who reported an increase in plant height, number of branches and number of bolls, boll weight with combined foliar application of K and MLE. Increase in number of pods per plant might be due to more availability of K and other nutrients form foliar application of MLE which contains growth promoting hormone i.e. zeatin that improved pod formation, these results are in line with the findings of Moyo *et al*. [73]. Exogenous application mineral elements improved the growth and quality of produce in maize crop [74].

Other yield contributing attributes like 100-grain weight, biological yield, grain yield and harvest index were increased by foliar application of K and MLE in both sowing dates but kabuli chickpea performed better in normal sowing than late sowing. Overall improvement in yield attributes in normal sown kabuli chickpea is because of favorable environmental conditions as compared to late sown conditions. These findings are quite similar with the results of Ganguly and Bhattacharya [75] who reported sowing time effects the growth and development of chickpea and reported decrease in different morpho-physiological characteristics with late sowing due to unfavorable climatic conditions. Mohammadnejad and Soltani [76] reported an increase in yield contributing attributes (100-grain weight, biological yield, harvest index and grain yield) in case of early planting. Significant increase in yield and yield attributes of chickpea were observed in case of early planting as compared to late sowing [77]. In case of foliar applied K and MLE our results are similar to Goud *et al*. [78] who reported an increase in yield and yield related attributes like 100-grain weight, biological yield and grain yield with the application of K in chickpea. Similar results were also reported by Ganga *et al*. [70] who stated that an increase in 100-seed weight, seeds per pod, biological yield and grain yield by K application. Regarding the foliar application of K and MLE, all yield related attributes were enhanced. Improved yield and yield attributes might be due to fact that there was more availability of nutrients, supply of K, growth hormone, various micronutrients, phytohormones, growth boosting substances (ascorbic acid, phenols and minerals), cytokinin and gibberellic acid from MLE [79]. Our results are in line with the findings of Chattha *et al*. [80] and Yasmeen *et al*. [81] who reported that an increase in grain weight and grain yield was recorded by the application of MLE. Moreover, Mathew [82] and Ahmad *et al*. [83] also attained better crop yield by the application of MLE. Our findings also corroborated the results of Afzal *et al*. [84] who found an improvement in yield of late sown wheat by the foliar application of 3% MLE at tillering and booting stage. Our findings are similar to the results of Yasmeen *et al*. [72] who reported increase in boll weight, biological yield and lint yield in case of combined foliar application of K and MLE in cotton. Application of organic fertilizer improve the fertility status of soil with enhanced productivity of crops under stress conditions [85].

An increase in chlorophyll contents was also observed in chickpea by combined application of K and MLE followed by sole foliar application of MLE under sowing regimes in the current study. It might be due the fact that foliar application of K and MLE enhanced the nutrient availability, photosynthetic efficiency, carbohydrate synthesis and translocation. A decrease in chlorophyll contents in late sowing is due to short growth period and unfavorable environmental conditions. Our results are in line with the findings of Xu and Huang [86] who reported the decrease in chlorophyll contents and many physiological damages due to late sowing because of unfavorable environmental conditions like terminal heat stress in cool season crops. Regarding the foliar applied K and MLE, findings of current study are in accordance with Azeem and Ahmad [87] who reported that leaf chlorophyll contents were increased in tomato by foliar application of sole MLE and in combination of K, Fe and B. Similar findings related to our study were also reported by Mona [88] who stated that foliar application of MLE increased chlorophyll contents in *Erusa vesicaria*. Increment in gas exchange attributes antioxidant activities by foliar application of sole MLE, K and MLE, might be due to the presence of different alellochemicals and various secondary metabolites like phenols, ascorbate [30] and zeatin [89]. Our results are in line with the findings of Mona [88] and Abdalla [90] who reported increase in transpiration rate and stomatal conductance by foliar application of MLE in *Erusa vesicaria*. The boost in proline contents is due to the fact that MLE and K increased different organic solutes like soluble proteins, free amino acids and soluble sugars that ameliorate the negative impact of climatic conditions in late sown conditions [91]. Our results regarding antioxidants’ activities confirmed the findings of Rady *et al*. [65] who reported that foliar application of MLE alone in combination with other nutrients can maintain water status and avoid membrane damage, activate plant defense system and increase antioxidant levels in plant. Jan *et al*. [92] also reported an increase in antioxidant enzymatic activities like superoxide dismutase, ascorbate peroxidase and catalase by foliar feeding of K in combination with biostimulants. Increase in protein and K contents in sole K, MLE and combined K with MLE might be due the enhanced availability and absorption of various minerals and nutrients present in MLE that augmented the source efficiency of leaves. Our results are in agreement with Anantharaj and Venkatesalu [93] who reported that proteins contents were increased by the use of MLE that boosted absorption and translocation of minerals and nutrients. Rehman *et al*. [29] also reported that application of plant growth promoters in combination with mineral elements improved the early growth, better establishment of seedlings and other yield contributing factors.

## Conclusion

Foliar applied MLE and K sole and in combination significantly affected growth, physiological, biochemical, quality and yield attributes of kabuli chickpea cultivated under normal and late sown conditions. However, combined foliar application of K and MLE showed maximum increase in growth, physiological, gas exchange, biochemical, enzymatic activities, yield and quality attributes of kabuli chickpea grown under normal and late sown conditions. Hence, it is concluded from the findings of current study that foliar application of K and MLE at flowering stage can be boost growth and yield of kabuli chickpea cultivated under normal and late sown conditions.
